# TSG Targeting KDM5A Affects Osteogenic Differentiation of Bone Mesenchymal Stem Cells Induced by Bone Morphogenetic Protein 2

**DOI:** 10.1155/2022/6472864

**Published:** 2022-01-25

**Authors:** Min Wei, Yi Jiang, Yuanqing Huang

**Affiliations:** School of Stomatology, Hunan University of Medicine, Huaihua, Hunan 418000, China

## Abstract

**Objectives:**

To investigate the effect of 2,3,5,4′-tetrahydroxystilbene-2-O-*β*-D-glucoside (TSG) on the osteogenic differentiation of bone marrow mesenchymal stem cells (BMSCs) and its molecular mechanism.

**Methods:**

After TSG treatment of rBMSCs, alkaline phosphatase (ALP) activity was compared between the drug treatment group and the control group. The effects of TSG on alkaline phosphatase positive cloning and mineralized nodule formation were also detected. Total mRNA and protein were extracted, and the effects of TSG on the expression levels of osteopontin (OPN), osteocalcin (OCN), Runt-related transcription factor 2 (Runx2), Osterix, and Col1a1 were detected by real-time fluorescence quantitative PCR. Western blotting was used to detect the inhibitory effect of TSG on KDM5A. BMSCs were transfected with small interfering RNA (siRNA) targeting KDM5A (si-KMD5A) and pcDNA3.1 KMD5A.

**Results:**

TSG significantly increased the activity of ALP, the number of alkaline phosphatase clones, and calcified nodule formation. The OPN, OCN, Runx2, and Osterix expression levels were significantly increased among the osteoblasts after TSG treatment. A mechanistic study showed that the effect of TSG is realized by inhibiting KDM5A.

**Conclusions:**

KDM5A signaling may be involved in the regulation of osteogenic differentiation of rBMSCs. TSG can promote osteogenic differentiation and maturation of rBMSCs at 0.1–50 *μ*mol/L. The mechanism of action was realized by inhibiting the expression of KDM5A.

## 1. Introduction

Osteoporosis (OP) is a metabolic bone disease characterized by reduced bone mass, damaged bone mass, and reduced bone strength, resulting in increased bone fragility and proneness to fracture. Osteoporosis is characterized by complexity, comprehensiveness, youth, and masculinity. Therefore, research on the etiology and pathogenesis of osteoporosis must have a new understanding and improvement. Bone marrow mesenchymal stem cells (BMSCs) are derived from bone marrow and have the function of self-renewal and multidifferentiation [1]. The osteogenic differentiation ability of BMSCs decreases with age [2, 3]. In osteoporosis patients, the proliferation and self-renewal capacity of MSCs are reduced, the number of apoptotic cells is increased, osteogenic differentiation is weakened, lipogenic differentiation is enhanced, and the regulation of multidirectional differentiation is disordered [4–6].

TSG is an active component of *Polygonum multiflorum* and has a wide range of biological activities [7–9]. Studies have shown that TSG has antiaging, antiatherosclerotic, antihyperlipidemic, antitumor, anti-inflammatory, free radical scavenging, liver protection, and other biological activities [10–14]. TSG has a wide application prospect.

Histone methylation modification is one of the most important aspects of epigenetic research. Histone methylation is dynamically regulated by histone methylase and histone demethylase. Histone lysine demethylase 5A (KDM5A) is an important member of the histone demethylase family. KDM5A can specifically remove dimethyl and trimethyl groups (H3K4me2/3) from the fourth lysine of histone H3, thereby mediating gene silencing and regulating cell function [15, 16]. KDM5A can directly or indirectly maintain tumor cell dryness, inhibit cell metabolism and differentiation, and promote the proliferation, metastasis, and drug resistance of tumor cells. Therefore, KDM5A is closely related to the occurrence and development of a variety of diseases and is expected to be a new potential target for the treatment of osteoporosis.

In this study, the effects of TSG on osteogenic differentiation and maturation as well as the regulation of the KDM5A signaling pathway were studied in rat rBMSCs, to provide potential targets and candidate compounds for the treatment of osteoporosis.

## 2. Methods

### 2.1. Isolation and Culture of Rat Bone Marrow Mesenchymal Stem Cells

Five rats (12 weeks old) were obtained from Vital River Laboratory Animal Technology Co., Ltd. (Beijing, China), and were anesthetized by intraperitoneal injection of 10 mg/kg phenobarbital sodium. In addition, the rats were killed by CO_2_ suffocation. Femur and tibia were rapidly separated under aseptic conditions and epiphyses were removed at both ends. DMEM/F12 culture medium was extracted with a 5 mL syringe to flush the bone marrow cavity until the liquid was clarified. The rinse solution was collected, blown with a micropipette, and left to stand for 5 min. The supernatant was centrifuged at 1000 r/min for 5 min, and the supernatant was discarded. The cells were resuspended in DMEM/F12 containing 10% FBS. After repeated blowing and counting, 10^4^ cells/cm^2^ were inoculated into a 6-well plate and cultured in an incubator at 37°C and 5% CO_2_. First liquid changed after 3 days. Cell growth was observed daily. After 80% of the adherent cells were fused, trypsin was used for digestion and subculture (this was the first generation P1). When cells passed P3, the inoculation densities of the 96-well plate, 24-well plate, and 6-well plate were 2 × 103, 2 × 105, and 4 × 105 cells/well, respectively. All experiments were performed at Hunan University of Medicine, and approval was obtained from the animal ethics committee of Hunan University of Medicine.

### 2.2. Induction of Bone Differentiation

When the P3 generation MSCs in each group reached 80%∼90% fusion, the digestive cells were digested. MSCs were inoculated into a six-well plate. After 24 h, the old culture medium was removed, and 2 mL of osteogenic induction liquid (bone morphogenetic protein 2) was added to each well. Liquid was exchanged every 3 days for 21 consecutive days. The treatment group was given TSG at concentrations of 1, 10, and 50 *μ*mol/L.

### 2.3. Cell Transfection

Small interfering RNA (siRNA) targeting KDM5A (si-KMD5A) and siRNA negative control (si-NC) were all obtained from Shanghai GenePharma Co., Ltd. (Shanghai, China). The cDNA encoding KMD5A was amplified by PCR and then ligated into the pcDNA3.1 (+) vector (Invitrogen). Cell transfection was performed using Lipofectamine 2000 (Invitrogen). After 48 h, the transfection efficiency was validated by RT-qPCR analysis.

### 2.4. Determination of Alkaline Phosphatase Activity

The cells were inoculated in 12-well plates and cultured for 24 h for osteogenesis induction. The treatment group was given 10 *μ*mol/L TSG, and the control group was given blank induction medium. The culture medium of both the administration group and the control group contained 1‰ DMSO. After 7 days, ALP histochemical staining was performed by the azo method. The solution was washed with PBS twice, fixed with 10% formaldehyde solution for 1 min, add matrix solution (Michaelis barbiturate-HCL buffer containing 0.1% *α*-naphthol sodium phosphate and solid blue RR salt, pH 8.9), and left to react within 30 min. When brown spots appeared, the matrix solution was discarded, washed with PBS, and fixed, and the results were photographed for preservation. The area, quantity, and gray level of CFU-FALP were scanned by Image-Pro Plus 6.0 software for statistical analysis.

### 2.5. Alizarin Red S Staining

The cells were inoculated in a 24-well plate. Osteogenic differentiation was induced after 24 h of culture. The administration group was given 10 *μ*mol/L TSG. The blank induction medium was added to the control group, and the culture medium in both the administration group and the control group contained 1‰ DMSO. The culture medium was discarded on day 12. The cells were washed with PBS twice and fixed with 10% formaldehyde for 5 min. Alizarin Red dye was added and incubated at 37°C for 1 h. The formation of mineralized nodules was observed. The results were saved by photography, and the area, quantity, and grayscale of mineralized nodules were scanned by Image-Pro Plus 6.0 software for statistical analysis.

### 2.6. QRT-PCR

The cells were inoculated in 6-well plates and cultured for 24 h for osteogenesis induction. The administration group was given 10 *μ*mol/L TSG, and the control group was supplemented with blank induction medium. Both the administration group and the control group contained 1‰ DMSO. Total RNA was extracted by the kit method, and its concentration and purity were determined by ultraviolet-visible spectrophotometry. The RNA concentration was adjusted to 1 *μ*g, and 1 *μ*L was taken as cDNA. Primers and SYBR Green reagent were added to the system. cDNA was amplified by a two-step method on a BIO-RAD CFX96 real-time quantitative PCR instrument. In the predenaturation stage, the reaction took place at 95°C for 10 min, with a cycle. The PCR stage was 40 cycles of reaction at 95°C for 15 s, 57°C for 30 s, and 72°C for 30 s. The mRNA expression of the target gene in the drug delivery group and the mRNA expression of the control group were obtained. Internal parameter sequence was as follows: GAPDH forward: TACCCACGGCAAGTTCAACG, reverse: CACCAGCATCACCCATTTG. The CT (cycle threshold) value was recorded using ΔΔ CT = (CT purpose gene-CT inside) treatment group−(CT purpose gene-CT inside) control, computing each group 2^−ΔΔCT^.

### 2.7. Western Blot

The cells were inoculated in 6-well plates and cultured for 24 h for osteogenesis induction. The treatment group was given TSG at concentrations of 1, 10, and 50 *μ*mol/L. The blank induction medium was added to the control group, and the culture medium in both the administration group and the control group contained 1‰ DMSO. After 3 days, the total protein was extracted from each well with 300 *μ*L cell lysate (containing PMSF 1 mmol/L). The protein concentration was detected by BCA method. Sample loading buffer containing bromophenol blue was added and denatured at 95°C for 5 min. After 12% SDS-PAGE electrophoresis, the protein was transferred to a PVDF membrane. The shaker was sealed with 5% skimmed milk powder at room temperature for 1 h. KDM5A primary antibody diluted with TBST (Abcam, dilution ratio: 1 : 1000) was added and left at 4°C overnight. The next day, the PVDF membrane was washed three times with TBST, and then horseradish peroxidase-labeled secondary antibody diluted with TBST was added. The cells were shaken at room temperature for 2 h. After washing the film 3 times, the gray value of the protein was detected by an exposure meter.

### 2.8. Statistical Analysis

The results are presented as the mean ± standard deviation. SPSS 16.0 software was used to process the data, and ANOVA was used to analyze and compare the differences between multiple groups. Student's *t*-test was used to analyze the comparison between the two groups. *P* < 0.05 was considered statistically significant.

## 3. Results

### 3.1. Effects of TSG on the Toxicity and Osteogenic Differentiation of Bone Marrow Mesenchymal Stem Cells (rBMSCs)

Figure 1(a) shows the molecular structure formula of TSG. To investigate the effects of TSG on BMSCs, we first analyzed the effects of different concentrations of TSG on cell proliferation. Experimental results showed that TSG did not affect cell proliferation (Figure 1(b)). Furthermore, we evaluated the effect of TSG on alkaline phosphatase in rBMSCs. Experimental results showed that an alkaline phosphatase activity-positive clone (CFU-FALP) could be formed in both the control group and administration group. After TSG treatment (1, 10, and 50 *μ*mol/L), the area, quantity, and relative gray level of CFU-FALP were higher than those of the control group, and the difference between the two groups was statistically significant (Figure 1(c)). Further experimental results showed that different concentrations of TSG increased ALP activity (Figure 1(d)) and presented a concentration-dependent effect. The influence of TSG on the formation of calcified nodules showed that both the control group and the TSG group formed calcified nodules after osteogenic induction of rBMSCs. After TSG treatment (1, 10, and 50 *μ*mol/L), the number of calcified nodules was greater than that of the control group. According to IPP 6.0 software analyses, the area, number, and relative grayscale of calcified nodules were higher than those of the control group, and the difference between the two groups was significant (Figures 1(e) and 1(f)). Furthermore, we examined the effect of TSG on osteogenic differentiation-related proteins. The results showed that TSG treatment at different concentrations upregulated the expression of OPN, OCN, Runx2, and Osterix (Figures 2(a)–2(d)).

### 3.2. Knockdown of KDM5A Promoted Osteogenic Differentiation of Bone Marrow Mesenchymal Stem Cells

Through experiments, we found that the expression of KDM5A was decreased during the osteogenic differentiation induced by BMP-2 (Figure 3(a)). Western blot results also showed that bMP-2 induction could inhibit the expression of KDM5A (Figure 3(b)). To further investigate the direct role of KDM5A in the osteogenesis of MSCs, we knocked down KDM5A in normal MSCs (Figure 4(a)). Alkaline phosphatase staining results showed that KDM5A knockdown promoted ALP activity under BMP-2-induced osteogenic differentiation (Figure 4(b)). Alizarin Red staining showed the knockdown of KDM5A, which significantly promoted bMP-2-induced mineralization deposition (Figure 4(c)). In addition, RT-PCR showed that KDM5A knockdown downregulated the expression levels of OPN, OCN, Runx2, Osterix, and Col1a1 (Figures 4(d)–4(h)). These results indicate that KDM5A negatively regulates osteoblast differentiation. Elevated KDM5A may be the cause of osteoporosis.

### 3.3. Influence of TSG on KDM5A Expression

Furthermore, we evaluated the effect of TSG on KDM5A expression. First, we treated primary rBMSCs with different concentrations of TSG. By real-time qPCR detection of KDM5A expression changes, 2^−ΔΔCT^ analysis of test results was performed with a relative quantitative method. The experimental results showed that, compared with the control group, the gene expression of KDM5A was significantly inhibited in the TSG group at different concentrations (Figure 5(a)). Western blot results were consistent with qRT-PCR results. Experimental results showed that TSG treatment could inhibit the protein expression of KDM5A (Figure 5(b)).

### 3.4. TSG Promotes Osteogenic Differentiation of Bone Mesenchymal Stem Cells by Targeting the Expression of KDM5A

To further investigate the direct effect of TSG on the osteogenesis of MSCs by inhibiting KDM5A, we overexpressed KDM5A in normal MSCs (Figure 6(a)). Alkaline phosphatase staining results showed that, under the osteogenic differentiation induced by BMP-2, overexpression of KDM5A inhibited the activity of ALP, while TSG treatment upregulated the activity of ALP (Figure 6(b)). Alizarin Red staining showed that overexpression of KDM5A significantly reduced BMP-2-induced mineralization deposition, while TSG treatment upregulated mineralization (Figure 6(c)). In addition, RT-PCR showed that KDM5A overexpression inhibited the expression of OPN, OCN, Runx2, Osterix, and Col1a1, while TSG treatment upregulated the expression of these genes (Figures 6(d)–6(h)). These results indicated that KDM5A inhibited osteoblast differentiation, while TSG could play a protective role by inhibiting the expression of KDM5A.

## 4. Discussion

BMSCs are derived from bone marrow and have the functions of self-renewal and multidifferentiation. They can differentiate into osteoblasts, adipocytes, myoblasts, chondroblasts, and nerve cells under certain conditions [1]. BMSCs can promote osteogenic differentiation and increase bone formation and strength. In recent years, the application of BMSCs in cell therapy for bone-related diseases has attracted great attention. BMSCs also show great application potential in bone tissue engineering [1, 17, 18]. The results showed that TSG could promote osteogenic differentiation and maturation of BMSCs and significantly improve ALP activity, ALP-positive clone formation, and calcified nodule formation. TSG can increase the expression of Runx2 and other genes, which are closely related to the osteogenic differentiation of cells.

In recent years, studies have shown that plant drugs have great potential in the prevention and treatment of osteoporosis. On the basis of traditional Chinese medicine formulations, several Chinese patent medicines against osteoporosis have been developed and improved. Wang et al. [19] summarized 12 randomized controlled trials of proprietary antiosteoporosis drugs and evaluated their effectiveness, including 1816 patients with osteoporosis. The results showed that all the herbal preparations significantly increased the lumbar spine bone density. A variety of flavonoid compounds have been shown to contribute significantly to bone formation at the cellular or animal levels, for example, icariin, genistein, resveratrol, and osthole [19–23]. Compared with traditional osteoporosis medicine, plant medicine has wide sources and few side effects [24, 25]. Therefore, it has great application development value. TSG is the main component of Polygonum multiflorum and has good water solubility [12, 13]. At the same time, it has antioxidant functions and scavenges free radicals. TSG also has a variety of biological regulatory effects, such as antiosteoporosis, vasodilation, and anticomplement activity. In this study, it was found that TSG promoted osteoblast differentiation not through the estrogen signaling pathway but by inhibiting the expression of KDM5A. We found that TSG can enhance the expression of the OPN, OCN, Runx2, and Osterix genes. Western blot analysis further proved that TSG treatment could reduce the protein expression level of KDM5A. The results show that TSG may promote the differentiation and maturation of BMSCs by regulating KDM5A signaling.

KDM5A is a histone demethylase that can specifically remove dimethyl and trimethyl groups (H3K4me2/me3) from the fourth lysine of histone H3, so it is also known as H3K4me2/3 demethylase [26–28]. KDM5A plays an important role in cell development and differentiation [29]. At present, the regulatory mechanism of KDM5A on cell differentiation is not very clear. Several studies have shown that KDM5A regulates cell differentiation mainly through indirect pathways. In mouse embryonic stem cells, KDM5A can synergistically affect Krüppel-like factor 4 (KLF4) to block the programming of pluripotent stem cell differentiation [30]. Furthermore, KDM5A maintained the desmethylation state of the core pluripotent transcription factor POU5F1, thereby inhibiting embryonic stem cell differentiation and maintaining cell dryness. In addition, KDM5A can also form a coinhibitory complex with a polycomb group (PcG) to jointly maintain cell dryness and inhibit cell differentiation [31].

This study also has deficiencies. The differentiation and maturation of BMSCs are a complex process, and whether other signaling molecules or other signaling pathways are involved in the TSG regulation of osteogenic differentiation of rBMSCs remains to be further studied.

## 5. Conclusion

In conclusion, KDM5A is involved in the regulation of osteogenic differentiation of MSCs. Inhibition of KDM5A promoted osteogenic differentiation of MSCs. TSG was added to MSC culture to promote differentiation and mineralization to osteoblasts without affecting cell proliferation. Experimental results confirmed that TSG can promote osteogenic differentiation. Further research on the specific mechanism of TSG and KDM5A in regulating MSC behavior will provide an experimental basis for gene-targeted therapy and drug cell therapy for OP.

## Figures and Tables

**Figure 1:** Effects of TSG on the toxicity and osteogenic differentiation of bone marrow mesenchymal stem cells (rBMSCs). (a) Display of TSG molecular structure. (b) rBMSCs were treated with TSG at different concentrations for 1∼2 days, and cell count CCK-8 was used to detect cytotoxic effects. (c) TSG treatment of rBMSCs for 1 week and alkaline phosphatase staining of rBMSCs with (d) TSG treatment for 1 week, and the activity of alkaline phosphatase was detected. (e) Mineralization of rBMSCs 2 weeks after TSG staining detection. (f) Statistical results of mineralization of rBMSCs 2 weeks after Alizarin Red S staining detection and TSG staining detection. Data were mean ± (S) D, ^*∗∗∗*^*P* < 0.001.

**Figure 2:** Effects of TSG on the expression of osteopontin (OPN), osteocalcin (OCN), Runt-related transcription factor 2 (Runx2), and Osterix. (a) Detection of OPN expression by qPCR. (b) OCN expression was detected by qPCR. (c) QPCR was used to detect Runx2 expression. (d) Detection of Osterix expression by qPCR. Data were mean ± (S) D, ^*∗*^*P* < 0.05, ^*∗∗*^*P* < 0.01, ^*∗∗∗*^*P* < 0.001.

**Figure 3:** KDM5A expression was downregulated under osteogenic differentiation induced by bone morphogenetic protein 2 (BMP-2). (a) The expression level of KDM5A was detected by qPCR. (b) Western blot detection of KDM5A expression. Data were mean ± (S) D, ^*∗*^*P* < 0.05, ^*∗∗*^*P* < 0.01.

**Figure 4:** Knockout of KDM5A promoted osteogenic differentiation of bone marrow mesenchymal stem cells. (a) qRT-PCR analysis of KDM5A expression in transfected MSCs. (b) Alkaline phosphatase staining and activity of MSCs with si-KDM5A were detected by ALP staining 7 days after osteogenesis induction. (c) Alizarin Red S staining was used to detect mineralized nodules of bone marrow mesenchymal stem cells after si-KDM5A. (d) qPCR was used to detect OPN expression in MSCs of si-KDM5A after osteogenesis induction. (e) qPCR detection of OCN expression in MSCs of si-KDM5A after osteogenesis induction. (f) qPCR was used to detect Runx2 expression in MSCs of si-KDM5A after osteogenesis induction. (g) qPCR was used to detect Osterix expression in MSCs of si-KDM5A after osteogenesis induction. (h) qPCR was used to detect Col1a1 expression in MSCs of si-KDM5A after osteogenesis induction. Data were mean ± (S) D, ^*∗*^*P* < 0.05, ^*∗∗*^*P* < 0.01, and ^*∗∗∗*^*P* < 0.001.

**Figure 5:** TSG treatment inhibits the expression of KDM5A. (a) The expression level of KDM5A was detected by qPCR. (b) Western blot detection of KDM5A expression. Data were mean ± (S) D, ^*∗∗*^*P* < 0.01 and ^*∗∗∗*^*P* < 0.001.

**Figure 6:** TSG promotes osteogenic differentiation of bone mesenchymal stem cells by targeting the expression of KDM5A. (a) qRT-PCR analysis of KDM5A expression in MSCs after different treatments. (b) Alkaline phosphatase activity was detected by ALP staining after osteogenic induction of MSCs in each group. (c) Alizarin Red S staining detection for mineralized nodules formed by bone marrow mesenchymal stem cells after staining detection in each group. (d) qPCR was used to detect the OPN expression of MSCs in each group after osteogenesis induction. (e) qPCR detection of OCN expression in MSCs treated in each group after osteogenesis induction. (f) qPCR was used to detect Runx2 expression in MSCs in each group after osteogenic induction. (g) qPCR was used to detect Osterix expression in MSCs treated in each group after osteogenic induction. (h) qPCR was used to detect the expression level of Col1a1 in MSCs in each group after osteogenic induction. MSC/V: cells treated with empty plasmid (vector). Data were mean ± (S) D, ^*∗*^*P* < 0.05, ^*∗∗*^*P* < 0.01, and ^*∗∗∗*^*P* < 0.001.

## Data Availability

The data used to support the findings of this study are available from the corresponding author upon request.
